# High-Fat Diet Promotes DSS-Induced Ulcerative Colitis by Downregulated FXR Expression through the TGFB Pathway

This article has been retracted.

**DOI:** 10.1155/2020/3516128

**Published:** 2020-09-26

**Authors:** Di Zhao, Chenwen Cai, Qiyi Chen, Shuang Jin, Bo Yang, Ning Li

**Affiliations:** ^1^Department of Colorectal Disease, Shanghai Tenth People's Hospital, Tongji University School of Medicine, Shanghai, China; ^2^Division of Gastroenterology and Hepatology, Key Laboratory of Gastroenterology and Hepatology, Ministry of Health, Shanghai Inflammatory Bowel Disease Research Center, Renji Hospital, School of Medicine, Shanghai Jiaotong University, Shanghai Institute of Digestive Disease, 145 Middle Shandong Road, Shanghai, China

## Abstract

Ulcerative colitis is one of the IBD which cause a chronic intestinal inflammation and dysfunctional of the mucosal barrier. For now, the incident of UC was steadily increased all over the world. It has become a novel independent risk factor of several severe diseases especially colon-rectal cancer. However, the etiology of UC was still obscure. Previous studies show that high-fat diet contributed to the pathogenesis of immune system dysregulation, and farnesoid X receptor (FXR) was also implicated in the pathogenesis of various inflammatory symptoms. Yet, their inner roles in the pathogenesis of UC have not been mentioned. In this study, we aim to investigate the role of FXR in UC. High-fat diet (HFD) promotes the progression of DSS-induced UC, shows an increasing secretion of bile acid in serum, and leads to a downregulation of FXR target genes (FXR*α*, Shp, and lbabp). Adding FXR agonist FexD rescues the phenotype induced by high-fat diet, whereas TGFBRI inhibitor SB431542 abrogates the restoration by FexD in DSS-induced UC mice. To further verify the relationship between the FXR and TGFB signaling pathway, we made a UC-HFD model in the Caco2 cell line. Results shows the same conclusion that FXR mitigate UC inflammation through a TGFB-dependent pathway. These results expand the role of FXR in ulcerative colitis and suggest that FXR activation may be considered a therapeutic strategy for UC.

## 1. Introduction

Ulcerative colitis (UC) is one of the inflammatory bowel diseases which result from mucosal immune system disorder and lead to chronic intestinal inflammation activation and structural dysfunction of the gastrointestinal tract [1]. Unlike Crohn's disease (CD) which can arise in any part of the gastrointestinal tract, UC mainly affects the colon and rectum [2]. The symptoms of UC are usually various, such as diarrhea, abdominal cramping, rectal pain, and blood in the stool. What is more, several studies illustrated that UC was an independent risk factor of colon-rectal cancer [3–5]. The incidence and prevalence of UC have recently steadily increased all over the world [6]. For now, its etiology remains elusive.

Previous studies reveal that the etiology and pathology of UC were multifactorial, primarily relate to the sensitivity of the intestine immunological stimuli, and result in the dysfunctional activation of mucosal immune system response [7]. Dysfunction of the mucosal barrier leads to the increasing intestine permeability and eventually triggering intestine inflammation involving the immune cell. Present therapeutic options such as the anti-TNF-*α* antibody infliximab, 5-aminosalicylic acids, and the corticosteroid prednisone were mainly used to inhibit the immune system and deliberate symptoms of patients [8].

While several conditions affect the UC-induced gastrointestinal problem, the role of high-fat diet in their course is often underestimated. According to research by Magro et al., increased intake of cholesterol and animal fat can increase the incidence of UC [9]. A study by Degirolamo et al. shows that HFDs result in equivalent upregulation in bile acids [10], which are potent inducers of UC, due to the hydrophobic nature of secondary bile acids lithocholic acid and deoxycholic acid promoting intestinal permeability effects [11, 12].

Transforming growth factor *β* proteins belong to a family of multifunctional polypeptides produced by multiple lymphoid and nonlymphoid cells [13]. UC is a kind of inflammatory bowel disease. TGFB1-3 have been reported as the keys in the regulation of immune cells. TGFB production is also related to the pathogenesis of colitis, which means the pathology of UC may be caused by the disorder of the TGFB pathway.

The farnesoid X receptor (FXR) is one of the nuclear receptors, in charge of nutrient uptake and elimination of toxic dietary components; mainly regulates the bile acid homeostasis through the gut-liver axis, and eventually maintains the essential aspects of the intestinal barrier [14, 15]. Although the relationship of HFDs, FXR, and UC has been investigated, the inner mechanisms remain obscure. Here, we suggest that FXR mitigate mucosal inflammation induced by HFDs through an activation of the TGFB pathway.

## 2. Results

### 2.1. HFDs Promote the Progression of DSS-Induced UC in Mouse

To understand the contribution of diets in the progression of UC, the mice were treated with 3.5% DSS for a week to develop symptoms of UC, for instance, diarrhea, rectal bleeding, and weight loss, and then, we maintain DSS-induced mice with a regular diet or HFD for 2 weeks. The daily change of body weight and DAI is shown in Figures 1(a) and 1(b); compared to the DSS-treated group, the body weight of the combination of DSS and HFD treatment group was significantly reduced from day 5 to day 14 (DSS vs. DSS+HFDs, 30.52 ± 0.42 vs. 22.73 ± 0.32, *P* < 0.01), and for DAI comparison, the dual treatment also makes the mice have significant increase among groups (DSS vs. DSS+HFDs, 2.33 ± 0.33 vs. 3.32 ± 0.30, *P* < 0.05).

Next, we assessed the total serum BAs in DSS-induced mice on ND and HFD; we found that there was approximately 3-fold increase between the DSS group and the DSS-HFD group (Figure 1(c)). In summary, HFDs promote the progression of DSS-induced UC in mouse.

### 2.2. FXR Mitigate the Tissue Damage in DSS-Induced Mice

FXR is one of the nuclear receptors that mainly regulate the bile acid homeostasis. The significant increase of bile acid in the DSS-HFD group gave us a clue that FXR may be involved in high-fat diet-exacerbated UC symptoms. So, we investigated the mRNA expression level of FXR*α*, Shp, and lbabp which were the target genes of FXR [16]. As showed in Figure 1(d), they all dramatically reduced in the DSS-treated plus high-fat diet group when compared to other groups. And in the DSS-treated-only group, they also significantly reduced with the vehicle group.

Next, we verify the function of FXR in mitigation of DSS-HFD-induced UC. We add the FXR agonist FexD to the daily diet of the DSS-HFD group. We found that FexD compensates for the UC phenotype caused by the dual treatment of HFD and DSS. DAI score and body weight loss were significantly decreased compared with the HFD-DSS group (Figures 2(a) and 2(b)). The concentration of bile acid in serum also markedly reduced with the treatment of FexD; however, it was to some extent blocked by the TGFBRI inhibitor SB431542 (Figure 2(c)). HE staining of the colon evaluated the histological changes. DSS treatment caused muscle thickening, crypt damage, and lymphocyte infiltration and HFD aggravates the symptoms; however, adding the FXR agonist FexD greatly reduced these symptoms (Figure 2(d)).

### 2.3. FXR Agonist Upregulated TGFB Signaling in DSS-HFD-Treated Mice

Since the TGFB pathway has been suggested to be related with the restoration of DSS-induced UC, we examined the key mediator to initiate the downstream TGF-beta signaling cascade-phosphorylated forms of TGFBRI and SMAD2 in the DSS-HFD group after FexD treatment by Western blot. Our data suggested that TGFBRI and SMAD2 were significantly upregulated.

To further testify whether the TGFB pathway is essential for FXR-related recovery of UC, we inhibit the TGFB signaling by using the TGFBRI inhibitor SB431542 in FexD-treated DSS-HFD mice. We found that SB431542 processing significantly offset the increase in TGFB signal in the FexD-treated DSS-HFD mouse colon, resulting in the failure of DAI reduction and reduced local inflammation (Figures 2(a)–2(d)). Western blot of the treated colon tissue protein shows that FexD can upregulate the expression of TGFBRI and the phosphorylated level of smad2.

And then, we exposed colonic epithelial cell (Caco2) to palmitic acid (PA) and TNF-*α*, to mimic HFD in UC situation. PA- and TNF-*α*-induced inflammation cytokine increase was dramatically inhibited by the FXR agonist FexD, and the TGFBRI inhibitor SB431542 (Selleck) can abrogate the influence of FexD. Therefore, these findings indicate that FXR activation can alleviate DSS-induced colitis by increasing TGFB signaling (Figure 3).

## 3. Material and Method

### 3.1. Animals and Treatment

6-week-old male C57BL/6 mice (18-20 g) were purchased from SLAC laboratory animal center; all mice are of SPF degree (Shanghai, China). For induction of ulcerative colitis, mice were fed with 3.5% DSS (MP Biomedicals) in their daily water with normal diet for a week and then, their diet was changed into high-fat diet provender which was purchased from XIETONG SHENGWU (XT10190019-1) containing 60% energy from fat for another 2 weeks. For FXR agonist experiments, fexaramine D was resolved in corn oil at the concentration of 50 mg/kg with or without the TGFBRI inhibitor SB431542 (Selleck) and then, oral gavage was used for 7 weeks of age DSS-treated mice on HFD for 2 weeks. DAI score and the histopathological scores of mice were assessed as described in the previous work [17].

### 3.2. Cell Culture and Treatment

Caco2 cell line was purchased from the American Type Culture Collection. It was cultured with the high-glucose DMEM (HyClone) supplemented with 10% FBS (Gibco), 100 *μ*g/ml of penicillin, and streptomycin at 37°C with 5% CO_2_ in a cell incubator. The cell was treated by 100 ng/ml TNF-*α*, 100 *μ*M palmitic acid, 10 *μ*M FexD, and 10 *μ*M SB431542 for 12 hours.

#### 3.2.1. Western Blot and Quantitative Real-Time PCR (qRT-PCR)

Treated mice colon tissue and cultured cells were freshly applied for total RNA extraction, using TRIzol reagent (Invitrogen) protocol. And then, quantitative real-time PCR was executed as described before. Briefly, 1 *μ*g of the total RNA was reverse transcribed into cDNA and then, the cDNA was conducted by using the SYBR system (Takara) following the manufacturer's instructions in an ABI 7500 real-time PCR machine. The mRNA expression level was calculated by the 2 − ΔΔCt method; the final values were normalized to the mRNA expression of GAPDH. The primers of gapdh, FXR*α*, Shp, and lbabp used for qRT-PCR are shown in Table 1. In performing Western blot, proteins were separated on different concentrations of SDS-PAGE gel (7.5%-10%), and then, the separated protein was transferred from gel to nitrocellulose (NC) membranes and blotted with respective primary antibodies, followed by appropriate secondary antibodies and then detected with ECL chemiluminescent system The primary antibodies used in this study were anti-*β*-actin (13E5, CST), p-Smad2 (D43B4, CST), and anti-TGFBRI (ab31013 Abcam).

### 3.3. Statistical Analysis

Data were showed as mean ± SD. Unpaired, two-tailed *E* Student's *t*-test was used to compare two groups of independent samples. Multiple comparison analysis was conducted by one-way ANOVA. SPSS Statistics version 20.0 software and GraphPad Prism 6 software were used for statistical analyses. All statistical tests with a *P* value of < 0.05 were considered significantly changed.

## 4. Discussion

In recent years, with changes in lifestyle and eating habits, the incidence of UC has gradually increased throughout the world and is closely related to the incidence of colorectal cancer. Studies [18] found that UC-related colorectal cancer only accounts for 1% to 2% of all colorectal cancers, but it accounts for 15% of the factors that cause death in UC patients. It can be considered that UC canceration is one of the main causes of death in UC patients. However, the etiology and pathogenesis are not yet clear. It is currently believed that changes in living environment, eating habits, immune system, genetics, and other factors may play an important role in the process of UC carcinogenesis.

High-fat diet is closely related to the onset of colitis and colorectal cancer. A recent research [19] proved that high-fat diet may increase the prevalence of UC in mice. Colitis mice who were given high-fat diet had increased local inflammation in the colon, indicating that high-fat diet may be a pathogenic factor of UC. The mechanism may be the metabolic decomposition of lipids in the digestive tract, such as secondary bile acid and hydrogen sulfide, which damage the intestinal microenvironment and induce inflammation of the colonic mucosa. The continuous accumulation of inflammation can lead to the occurrence of dysplasia and even cancer. High-fat diet is the main cause of obesity, and obesity is considered by most researchers as a “low-grade inflammation state.” Obesity-related inflammation plays an important role in the occurrence and development of cancer [20]. At present, there is a lack of relevant experimental and clinical studies on the effect of high-fat diet on UC cancer.

IL-6 is a kind of multipotency cytokine, which combines with receptors to form IL-6/IL-6R/gpl30 complex for signal transduction, inducing activation of transcription activator 3 and then exerting its biological function. Its main biological functions include regulating immune response and hematopoietic system, inducing acute-phase proteins and regulating tumor growth. In inflammatory bowel disease, whether it is Crohn's disease or UC, the CD4+ T cells that maintain chronic inflammation of the large intestine mainly rely on the antiapoptotic effect of IL-6, which is a core cytokine in the development of inflammatory bowel disease. In the gradual progress of inflammatory bowel disease and the eventual evolution of tumors, IL-6 not only helps tumor factors and promotes the occurrence of abnormal cells but also has an antiapoptotic effect on T cells and tumor cells [21]. Studies [22] have confirmed that blocking antibody-mediated IL-6 signaling can delay the formation of UC-related colorectal cancer induced by chemical carcinogens.

UC is a recurring disease. The onset and remission period vary in length. The recurrent inflammation leads to atypical hyperplasia of the intestinal mucosa and even cancer. It is difficult to collect multiple cycles of clinical cases. The main research method is to establish the corresponding animal model. This experiment proves that DSS-induced colitis is similar to human colon lesions. Colon pathology can show erosion and ulcer formation and a large number of inflammatory cell infiltration, and the lesions are confined to the mucosa and submucosa.

As an important immunomodulatory factor, TNF-*α* has a strong proinflammatory effect and is produced and released by immune cells and macrophages. TNF-*α* can further activate NF-*κ*B; stimulate the expression of proinflammatory factors IL-1, IL-6, IL-8, and IFN-*γ*; inhibit the expression of IL-10; promote inflammation; increase the permeability of epithelial cells; and initiate cytotoxicity, apoptosis, and acute phase reaction, which in turn causes intestinal mucosal damage [23].

In summary, our study demonstrated that FXR mitigate UC inflammation through a TGFB-dependent pathway. These results expand the role of FXR in ulcerative colitis and suggest that FXR activation may be considered a therapeutic strategy for UC.

## Figures and Tables

**Figure 1:** High-fat diet aggravates UC progression in a DSS-induced mouse model: (a) body weight change in mice on the treatment with DSS and HFD for 2 weeks; (b) DAI score change in mouse treatment with DSS and HFD for 2 weeks; (c) total bile acid concentration of serum in three experiment groups, respectively; (d) total RNA was extracted from the control group, DSS group, and DSS combination with HFD-treated colon to investigate the mRNA expression level of FXR*α*, Shp, and lbabp which were the target genes of FXR. ^∗^*P* < 0.05, ^∗∗^*P* < 0.01, and ^∗∗∗^*P* < 0.001 and *n* = 6 for each group.

**Figure 2:** FXR extenuate the tissue damage in DSS-induced mice: (a) body weight change in mice on combination treatment with DSS, HFD, FexD, and TGFBRI inhibitor SB431542 (Selleck) for 2 weeks; (b) DAI score change in mice on combination treatment with DSS, HFD, FexD, and TGFBRI inhibitor SB431542 for 2 weeks; (c) total bile acid concentration of serum in four experiment groups, respectively. ^∗^*P* < 0.05, ^∗∗^*P* < 0.01, and ^∗∗∗^*P* < 0.001 and *n* = 6 for each group; (d) representative images of five groups' colonic tissue stained with hematoxylin and eosin (H&E; upper) are shown. The bar represents 50 *μ*m and 20 *μ*m.

**Figure 3:** FXR extenuate the tissue damage in DSS-induced mice in a TGFB signaling-dependent way: (a) Western blot detects the TGFBRI and p-smad2 protein expression level in mouse colon on combination treatment with DSS, HFD, FexD, and TGFBRI inhibitor SB431542 for 2 weeks; (b) Western blot detects the TGFBRI and p-smad2 protein expression level in Caco2 cell line on combination treatment with TNF-*α*, PA, FexD, and TGFBRI inhibitor SB431542 for 12 hours; (c–f) RNA was isolated to assess the mRNA levels of proinflammatory cytokines (TNF-*α*, IL-6, IL-1*β*, and IL-8) in four different treatments by qRT-PCR. ^∗^*P* < 0.05, ^∗∗^*P* < 0.01, and ^∗∗∗^*P* < 0.001 and *n* = 3 for each group.

**Table 1:** The sequence of qRT-PCR primers.

qRT-PCR primer	Forward (5′-3′)	Reverse (5′-3′)
GAPDH (mouse)	AGGTCGGTGTGAACGGATTTG	GGGGTCGTTGATGGCAACA
FXR*α* (mouse)	GCACGCTGATCAGACAGCTA	CAGGAGGGTCTGTTGGTCTG
Shp (mouse)	GTACCTGAAGGGCACGATCC	GTGAAGTCTTGGAGCCCTGGT
lbabp (mouse)	CACCATTGGCAAAGAATGTG	AACTTGTCACCCACGACCTC
GAPDH (human)	GGAGCGAGATCCCTCCAAAAT	GGCTGTTGTCATACTTCTCATG
TNF-*α* (human)	CACATCTCCCAACACCTTAACTT	CCTCTCTCTAATCAGCCCTCTG
IL-6 (human)	ACTCACCTCTTCAGAACGAATTG	CCATCTTTGGAAGGTTCAGGTTG
IL-1*β* (human)	ATGATGGCTTATTACAGTGGCAA	GTCGGAGATTCGTAGCTGGA
IL-8 (human)	ACTCCAAACCTTTCCACC	CTTCTCCACAACCCTCTG

## Data Availability

The data related with our results can be provided when they are required.
